# The Impact of Tax Reduction and Fee Reduction Based on Big Data Algorithm on the High-Quality Development of the Real Economy under the Action of Coupling Effect or Substitution Effect

This article has been retracted.

**DOI:** 10.1155/2022/2828687

**Published:** 2022-08-10

**Authors:** Haiyan Zhang

**Affiliations:** Shool of Business, Zhengzhou University of Industrial Technology, Xinzheng 451100, Henan, China

## Abstract

The basic idea of the mass of medical growth is to adhere to local market price thinking with a Chinese touch and follow the development policy of “quality first, efficiency first.” It insists on properly handling a series of important relationships betwixt socialism and market economy, the first to drive the rich later, the government and the market, equality and efficiency, short-term growth and long-term development, China and the international economy, ecology and growth of the region. Under the guidance of the qualitative thinking theory, it combines the strategic goals of China's economic qualitative development and actively draws on the research results of other countries. It uses big data algorithms to focus on the impact of qualitative development on tax and income reduction in the real economy. It conducts research experiments on the impact of tax reduction and fee reduction based on big data algorithms on the top-notch growth of the real economy. Its experimental data show that: in 2018, the share of primary, tertiary, and primary sector in China's dimensional economy top-notch growth coordination index was 7.2%, 40.7%, and 52.2%, respectively. Its contribution rate to economic growth was 4.2%, 36.1%, and 59.7%, respectively. From these data, it can be concluded that the top-notch growth of the real economy is getting better and better under the influence of tax reduction and fee reduction by big data algorithms.

## 1. Introduction

The real economy is the foundation of cultural growth and the foundation of the healthy development of the national economy. However, many developed countries in Europe and America gradually give priority to the development of virtual economy. This has led to the continuous decline of the real economy, while the virtual economy is growing at an increasingly faster rate. It forms the phenomenon of economic transfer from physical to virtual. Statements such as “the real economy is the capital of the country,” “the strength of the country depends on the real economy,” and “promoting the development of the real economy” have been repeated in many important speeches by the Chinese general secretary. All these claims reflect the importance of the real economy to economic development. The real economy is the foundation to reach top grade status. If solid economy cannot achieve top-notch growth, it will be difficult for the economy to reach top grade status. However, the real economy is facing pressures such as weak innovation capability and increased resource and environmental constraints. It urgently needs to complete the transformation from quantity to quality. Effectively promoting the high-quality development of the real economy will play a catalytic role in deepening the supply-side structural reform. It is the focus of building a modern economic system and solving structural imbalances. It is also an important part of building a modern industrial system with coordinated development.

The real economy is lagging behind in the development process, and there are many problems such as insufficient growth rate, weak innovation ability, and resource and environmental constraints. Therefore, it is imperative to enhance the growth quality of our true market economy. At present, most of the literature on quality development focuses on the importance of economic quality development, the establishment the index of good quality growth of system, and the methods to promote the quality the growth of economy. It is necessary to establish a real economy quality development index system based on China's five major development concepts and use measurable indicators to determine the quality development level to reach top grade status, which will enrich the research content of quality development.

This paper studies top grade solid body structure construction on the basis of tax reduction and fee reduction of big data algorithms under the coupling effect or substitution effect. The quality index system for the development of the real economy is based on five aspects: creative growth, harmonious global scale, open economy, green culture, and the common development of the real economy. In the construction of the index system, it innovatively uses the degree of coordination between traditional industries and strategic emerging industries as an index to measure the coordinated development of the real economy. This makes the content of the coordination of the market real economy more comprehensive and richer. The index is to measure the quality of the market real economy and analyze the changes in the index and subindices of the quality of the market real economy view from the angle of time series. It found defects and shortcomings in the top-level economy development in real life. It complements the shortcomings of development, thereby providing new ideas for the top-level economy development in real life.

## 2. Related Work

This paper studies the impact of top-notch growth of the real economy, and these studies can be fully applied to research in this field. Ankargren et al. described financial variables constructed to correspond to various channels in the transmission mechanism [1]. Dybka et al. studied the transmission of aggregate capital buffer shocks to lending, prices and economic activity in Poland during the period 2002–2015 using multivariate time series techniques [2]. Celebi studied PDA in terms of computational intensity, feasibility of statistical inference, and wider application areas to improve the measurement of the impact of Brexit on the real economy [3]. Grassetti et al. studied discrete-time dynamic models with four variables and delays. It describes the interaction between the three-sector real economy and the financial market with four assets [4]. Prianyshnykova and Hudenko highlighted the financial and economic necessity and semantics of practical approaches for countries to overcome the negative impacts of the COVID-19 pandemic [5]. These approaches provide some inputs for our review, but given the brief length of time and low panel size of the studies in question, they have not been recognized by the public. Based on big data algorithms, we reviewed the following relevant materials to study the impact of tax reduction and fee reduction on the top-notch growth of the real economy. Dai and Ma studied the use of network information technology in big data in extremely large information systems. They quickly processed and analyzed these huge data information [6]. Lingam and Sudhakara provided parallel clustering algorithms mainly based on parallel programming. MapReduce is one of the most commonly used frameworks for this purpose. And it is highly valued for its flexibility, fault tolerance, and ease of programming [7]. Pradeep and Naveen believed that with the rapid development of information technologies such as the Internet and the Internet of Things, big data usually exists in cyberspace in the form of data streams [8]. Goodarzian et al. believed that big data (BD) approaches have had a significant impact on the development and expansion of supply chain network management and design [9]. Tchapga et al. described how these algos can be adapted to big data structures applying the Spark interface. He presented a further work flow for taxonomy based on watched optimal algorithms, support vector mechanisms, and deep study [10]. Li et al. proposed a basketball training algorithm utilizing big data and IoT. They proposed algorithm used continuous video motion features, trajectory features, and contextual information from key figures for gesture recognition [11].

## 3. The Impact of Tax Reduction and Fee Reduction of Big Data Algorithms on the High-Quality Development of the Real Economy under the Coupling Effect or Substitution Effect

China's economic development has entered a new stage, which requires higher quality and efficiency. The corresponding theoretical research, practical research, institutional research, and countermeasure research are obviously lagging behind, which does not meet the requirements of top-notch growth of the national economy in the new era. It improves the process of top-notch growth of the real economy by studying the impact of tax reduction and fee reduction of big data algorithms on the top-notch growth of the real economy under the coupling effect or substitution effect.

### 3.1. Big Data Algorithm under Coupling Effect or Substitution Effect

Interaction force is another word for mutual aid effect. In group psychology, the interaction of two or more entities in a cluster is a common reaction a force multiplier. In fact, the circular effect is also a binding effect, which only in a more specific form.

Substitution works by saying that earnings per place of time improve when the price tag does increases. Workers would rather sacrifice their free time in order to earn more money. The income effect means that when the wage rate increases, workers can earn the same income in less time. When the replacement function is wider than the wage impact, the salary growth increases and runs upward to the right. When the earning role is much higher, the substitute role growth reduces labor supply, which bends the labor supply curve backwards.

Data mining processing mainly includes data classification, frequent set mining, and data clustering. Data classification is a supervised knowledge learning method. Frequent set mining is a technique for discovering valuable associations between data items in a dataset. As one of the hot topics in the field of data mining, data clustering is also one of the basic methods in data analysis [12].

As an important unsupervised identification process, clustering has been widely used and studied. It can be used as a preprocessing before other data mining algorithms run, and it can be used alone to discover valid information in the database. Clustering is the process of dividing things into different categories according to certain rules and requirements. It divides the dataset into multiple categories according to a certain metric, so that the data within the same category are as similar as possible, and the data between different categories are as dissimilar as possible. According to whether the category of data points in the clustering process is unique, the clustering algorithm can be divided into soft clustering and hard clustering. Soft clustering can also be called fuzzy clustering.

Hard clustering can be described in mathematical language as follows:

(1) $$\begin{array}{c} M=\left\{m_{1},m_{2},\ldots ,m_{y}\right\}\in R^{y\times d}. \end{array}$$

It represents a given dataset, and the *i*th data point is represented by:

(2) $$\begin{array}{c} m_{i}\left(i=1,2,\ldots ,y\right). \end{array}$$

It sets the dataset *M* can be divided into *z* categories, namely,

(3) $$\begin{array}{c} C=\left\{C_{1},C_{2},\ldots ,C_{k}\right\}\left(z\leq y\right). \end{array}$$

Then, each category *C*_*i*_ should be satisfied, and each category must contain data points, as shown in the following formula:

(4) $$\begin{array}{c} C_{i}\neq \varphi ,\;\left(i=1,2,\ldots ,z\right). \end{array}$$

Each data point belongs to one and only one category of data, as shown in the following formula:

(5) $$\begin{array}{c} C_{i}\cap C_{j}=\varphi ,\;\left(1\leq i\neq j\leq z\right). \end{array}$$

The sum of all categories is the entire dataset as follows:

(6) $$\begin{array}{c} U_{i=1}^{z}C_{i}=M. \end{array}$$

The membership function *u*_*ij*_ represents the degree of membership of the point *x*_*j*_ to the cluster *c*_*i*_, and the formula is as follows:

(7) $$\begin{array}{c} m_{j}\left(j=1,2,\ldots ,y\right),\\ C_{i}\left(i=1,2,\ldots ,z\right). \end{array}$$

When *u*_*ij*_=1, it means *m*_*j*_∈*C*_*i*_. If *u*_*ij*_=0, then *m*_*j*_∉*C*_*i*_, that is, the membership function:

(8) $$\begin{array}{c} u_{ij}\in \left\{0,1\right\}. \end{array}$$

It is a binary function and satisfies:

(9) $$\begin{array}{c} \sum_{i=1}^{z}u_{ij}=1,\;\forall j,\\ 0<\sum_{j=1}^{y}u_{ij}<y,\;\forall i. \end{array}$$

However, in the complex real life, there are still some vague and imprecisely defined objects to be identified. Therefore, the introduction of fuzzy theory into clustering can describe the classification of such objects in a more specific and detailed manner, which results in fuzzy clustering. The class assignment of data points in fuzzy clustering is not unique. A data point can belong to several categories at the same time [13]. The introduction of fuzzy theory not only does not bring difficulties to knowledge discovery and learning but makes information exchange more convenient and easier to understand. The process of cluster analysis is shown in Figure 1:

Classical cluster analysis includes the following steps: (1) Data preparation: it includes feature normalization and dimensionality reduction; (2) Feature selection: it selects the effective features useful to the algorithm from all the features in the dataset. These effective features can make the values of samples of the same category close, while the values of samples of different categories are different; (3) Feature extraction: it forms new and more meaningful features through some transformations of the selected features; (4) Clustering: it chooses a similarity measure appropriate to the feature type or a distance function to measure the closeness between data points; (5) Evaluation and analysis of clustering results: it uses the evaluation index to evaluate the validity of the clustering results and makes a reasonable explanation based on the realistic background [14].

In recent years, big data processing frameworks have emerged. Nowadays, whether it is enterprises, governments, or schools, big data processing frameworks are gradually replacing the old technical computing frameworks. Hadoop is an application platform that stores and can process large amounts of data. It is open-source, free, and widely used software from the Apache Software Foundation. The Spark architecture diagram is shown in Figure 2:

Spark has extremely high compatibility, and it can be easily integrated with other open-source software. Spark does not necessarily rely on third-party resource management and scheduling systems but implements the standalone mode as its own internal scheduling framework. It also provides tools to deploy standalone Spark clusters in EC2, making Spark easy to deploy and use [15].

The concept of data mining was first mentioned at the 1995 American Computer Annual Conference. Mining data points to the below referencing process extracting knowledge and information from incomplete, massive, fuzzy, noisy, and random data. These data are not known in advance and are indirect but potentially useful. The process of extracting knowledge from data is an important form of data mining. It is also known as Knowledge Discovery Process (KDD) in Database and Knowledge Discovery Process, Data Mining Process, etc. It can be used in its process to detect relationships between concepts/classes, classification, anomaly analysis, similarity analysis, description and trend analysis, and visualization of results. Therefore, data mining can be understood as a database-based search process. This search refers to the exploration and organization of large amounts of data. Its purpose is to find out valuable hidden events and information. The schematic diagram of the KDD process is shown in Figure 3:

As can be seen from the figure, the main stages of KDD consist of the following parts: (1) Data cleaning: it removes noise or irrelevant data from the source data. (2) Data preprocessing: it mainly refers to data preprocessing, including data integration and transformation. This step can be understood as integration, integrating data suitable for data mining. (3) Data mining: according to the requirements of the subject, it proposes mining tasks and important steps. It just uses tools to find regular things in a large amount of data, that is, data pattern mining. (4) Data representation: that is, the visualization of a graph or table of extracted information [16].

The data mining analysis framework includes four stages: “proposing research questions,” “data preparation,” “data mining,” and “model analysis.” The data mining analysis framework is shown in Figure 4:

It analyzes and explores data from big data in an automatic way to discover potentially valuable information; carries out a series of exploration and repetition processes; and continuously circulates, corrects, and draws conclusions. It starts with the proposed research question first. The content and format of data preparation is determined based on the problem frame and assumptions. In the data preparation phase, it first summarizes the characteristics of the data. Then, the research results are deduced by using the built mining model, which finally analyzes the deduction results and tests the validity of data mining [17].

### 3.2. Tax Reduction and Fee Reduction

After the subprime mortgage crisis in 2008, China put forward the focus of fiscal work to implement structural tax cuts. It uses a panel data multiple linear regression model to test how tax and fee reductions will affect the top-notch growth of the real economy. Specifically, in order to test H1, it adopts the following algorithm as the regression model:

(10) $$\begin{array}{c} EVX_{it}=\beta_{0}+\beta_{1}{\text{Fin}}_{it}+\delta {\text{controal}}_{it}+\varepsilon_{it}. \end{array}$$

In order to test H2, the regression model formula is used as follows:

(11) $$\begin{array}{c} EVX_{it}=\beta_{0}+\beta_{1}Txa_{it}+\delta controal_{it}+\varepsilon_{it} \end{array}$$

In order to test H3, the regression model formula is as follows:

(12) $$\begin{array}{c} EVX_{it}=\beta_{0}+\beta_{1}{\text{Fin}}_{it}+\beta_{2}{\text{Fin}}_{it}Txa_{it}+\beta_{3}Txa_{it}+\delta {\text{controal}}_{it}+\varepsilon_{it}. \end{array}$$

With the trend of economic financialization and the phenomenon of “departing from the real to the virtual” in the real industry, the high-risk and high-return virtual economy has gradually become more attractive to real enterprises. The reduction of funds for investment and operation of the main business leads to the decline of core competitiveness. This will inevitably bring greater risks to enterprises and reduce the sustainable development of the manufacturing industry. The key to the sustained value growth of the real industry lies in maintaining the stable development of the main business. Therefore, manufacturing state-owned enterprises with low earnings persistence cannot make full use of their resources, resulting in a decline in the real economy [18].

To test this claim, it constructs a mediation effect model. Among them, Croa is the continuity of earnings, which is measured by the main business profit/average total assets. Higher values indicate better earnings persistence. The specific model is as follows:

(13) $$\begin{array}{c} EVB_{it}=\beta_{0}+\beta_{1}{\text{Fin}}_{it}+\delta {\text{controal}}_{it}+\varepsilon_{it},\\ {\text{Croa}}_{it}=\beta_{0}+\beta_{1}{\text{Fin}}_{it}+\delta {\text{controal}}_{it}+\varepsilon_{it},\\ EVB_{it}=\beta_{0}+\beta_{1}{\text{Fin}}_{it}+\beta_{2}{\text{Croa}}_{it}+\delta {\text{controal}}_{it}+\varepsilon_{it}. \end{array}$$

Financialization has a “substitution” effect on real enterprises, and the transfer of capital to financial markets deprives companies of the means to innovate, thereby weakening the foundation for innovation. The return on financial investment is higher than the return on actual investment, and the excess return on financial investment is a strong disincentive. In addition, due to the complex principal–agent relationship in Chinese enterprises, managers focus more on financial investment rather than business innovation to achieve short-term operating results. It enables SOEs to raise capital through short-term, reversible financial investments rather than investing in long-term, irreversible investments. Innovative behavior can bring abundant funds for the future development of enterprises and obtain higher product leadership. It ensures that the enterprise has a sustainable competitive advantage in the process of development, thereby further enhancing the value of the enterprise. Based on this, it proposes a path to inhibit manufacturing state-owned enterprises by reducing innovation input [19].

To test this pathway, a mediation effect model was constructed. Among them, R&D is innovation input, which is measured by R&D expenditure/operating income. The specific formula is as follows:

(14) $$\begin{array}{c} EVZ_{it}=\beta_{0}+\beta_{1}{\text{Fin}}_{it}+\delta {\text{controal}}_{it}+\varepsilon_{it},\\ R\wedge D_{it}=\beta_{0}+\beta_{1}{\text{Fin}}_{it}+\delta {\text{controal}}_{it}+\varepsilon_{it},\\ EVZ_{it}=\beta_{0}+\beta_{1}{\text{Fin}}_{it}+\beta_{2}R\wedge D_{it}+\delta {\text{controal}}_{it}+\varepsilon_{it}. \end{array}$$

According to the formula calculation and analysis, it can be concluded that innovation input is an intermediary variable between finance and production and has a partial intermediary effect. That is, lower innovation inputs hinder productive activities.

Since China proposed structural tax cuts in 2008, tax cuts have been continuously updated, ranging from structural tax cuts to the current parallel tax cuts and tax cuts. During the implementation of the tax reduction policy, it can be seen that the state attaches more and more importance to tax reduction, and the influence of tax reduction is increasing [20].

At the 2019 National People's Congress, the Prime Minister emphasized that “reducing taxes and fees” is one of the main tasks for 2019. Efforts are needed to reduce corporate tax burdens and improve market conditions. The need was also underlined in the Chinese Party's 19th Congress report and continue to carry out the work of reducing overcapacity, reducing costs, and making up for shortcomings. It is necessary to further streamline administration and delegate power, reduce taxes and fees.

Data from the National Bureau of Statistics show that since the founding of New China, private enterprises have developed rapidly. In 2018, amount of small private-owned factories amounts to 65.794 million, accounting for 95% of the market units. Private enterprises have become an important pillar of China's economy, contributing up to 60% of China's GDP and generating more than 50% of tax revenue. According to the analysis information of the top 500 private enterprises in 2017, the after-tax net profit of the top 500 private enterprises in 2017 was about 1.13 trillion yuan, with an increase of 35.5% over 17 years ago. Its import and export volume reached 27.8 trillion yuan, accounting for 5.51% of China's total exports. For their part alone, the real data are strong evidence of the role private enterprises that play in China's economic growth. In terms of taxation, in 2017, the top 500 private enterprises paid 7.6% of the total tax revenue, and the tax amount reached 1.03 trillion yuan. Private enterprises have become a force that cannot be ignored in national taxation.

The theoretical significance of tax reduction and fee reduction is that under the circumstance of effectively reducing taxes and fees for enterprises, enterprises have abundant funds, and the further enhancement of liquidity will definitely increase the enthusiasm of enterprises to invest [21, 22]. After the liquidity of funds is fully mobilized, the production capacity of the real economy will be greatly improved. However, after the level of economic development is improved, the overall economic scale will inevitably expand. This expands the tax base, and the total tax revenue will rise instead of falling.

The policy significance of tax reduction and fee the downsizing is to minimize federal pressure of enterprises, which may play a role in promoting enterprises to deleverage. The reduction of leverage will further increase the liquidity of enterprises and finally achieve a boom in production and sales.

The theoretical and policy significance of reducing taxes and fees will help to greatly improve the quality and level of China's economic development. At the same time, it will accelerate the transformation of China's economic structure and achieve long-term and stable economic growth. At the same time, it will also bring an increase in per capita disposable income, promote the common prosperity of the people, greatly increase the level of consumption, and stimulate the overall economic growth [23, 24].

China's macro tax burden has been high for a long time. For this reason, whether it is the era of the “troika” of demand-driven economy, or since the supply-side structural reform, tax reduction and fee reduction are consistent practices in the formulation and implementation of China's tax policies. Especially after the outbreak of the economic crisis in 2008, China has formulated a large number of policies in reducing taxes and fees.

Macroeconomic tax burden represents the share of tax revenue in a country's GDP in a given period. The overall tax burden of a country can be illustrated by the macroeconomic tax burden. This is the most important indicator to study a country's tax burden. After studying and comparing the tax burden levels of other countries, Chinese experts believe that China's macro tax burden, especially corporate tax burden, is obviously at a high level internationally. The proportion of tax revenue to GDP is shown in Figure 5:

As can be seen from Figure 5, China's macro tax burden changes from 1999 to 2016. It can be seen that there has been an almost constant upward trend. The proportion of China's tax revenue to GDP has risen from 12.5% in 1999 to its highest point since 2012, with 19%. Although there has been a slight downward trend since then, it has risen to a level of about 50% more than in 1999. The annual growth rate of macro tax burden has reached an astonishing 16%. In recent years, China's tax pain index has been at the top of the list published by the famous Forbes magazine in the United States.

### 3.3. High-Quality Development of the Real Economy

The concept of “high-quality economic development” is a multi-level, cross-government, and cross-system economic category system. It includes concepts and categories such as development, economy, economic development, quality, economic quality, and economic development quality. These concepts and categories require accurate, comprehensive, scientific, and clear definitions and connotations so that relevant theoretical and empirical research can be built on rigorous scientific concepts and categories. It involves the influencing factors of the corresponding economic variables of a single economic unit and emphasizes how the price mechanism solves specific resource allocation problems.

Economics is a concept with several levels and stages. From a vertical perspective, economics has layers, which can be divided into macroeconomics, mesoeconomics, and microeconomics [25]. Macroeconomics refers to the entire economy, involving the efficient allocation of resources, the relationship between relevant aggregates, and the laws of development and change. Mesoeconomics deals with structural and coordinated economic issues such as sectoral, urban, rural, regional, and international economies. Microeconomics deals with the economic behavior of individual economies. Horizontally, the economy is divided into different stages, which can be subdivided into stages of production, exchange, distribution, and consumption. Each stage contains the micro, meso, and macro aspects of the economy. For example, the production stage mainly includes supply and demand, business innovation, industrial structure, and macroeconomic policies.

“Development” is an important term referring to human activity and the growth and evolution of various organisms. The definition of the term “development” is as follows: development refers to “the change of things from small to large, from simple to complex, and from low level to high level.” Development is a dynamic term that refers to a process of change from quantitative to qualitative, and from low level to high level. It is a holistic term that expresses a multidimensional state of change. It includes degree, quantity, quality, level, structure, and so on. It is a positive, complimenting word that includes progress, civilization, values, and so on.

“Quality” is a semantically important term that denotes the level and scope of human activity and its consequences. The concept of “quality” has two levels: first, it conforms to specifications, that is, the degree to which products manufactured and services provided conform to a certain specification, usually measured by a set of data. Second, it meets customer needs, that is, the degree to which a product or service meets customer expectations in terms of use and consumption. The concept of quality is essentially a value assessment. It can be described as “good” or “bad” and “better” or “worse”.

“Quality of economic development” is a dynamic and multidimensional concept. It refers to the degree of development and sustainability of a country or region in terms of economic aggregate, economic efficiency, economic structure, economic distribution, economic system, and economic environment. It includes the degree of growth of the total economic volume, the degree of improvement of economic efficiency, the degree of optimization of economic structure, the degree of fairness of economic development, and the degree of sustainability of economic development. From the overall indicators of top-notch growth of the real economy, the trend of top-notch growth of the real economy in China over the years is shown in Figure 6:

It is evident from the plot of the top-notch growth that level of China's real economy has been steadily rising since 2004, and the rate of increase has increased after 2015. It has implemented a series of policies that are beneficial to enterprises and social innovation activities and cultivated a soil for innovation. This shows that the top-notch growth level of China's real economy in recent years is generally in good shape. From the perspective of innovation indicators of top-notch growth of the real economy, the trend of innovation indicators of the real economy in China over the years is shown in Figure 7:

From the figure, the innovation index of top-notch growth of China's real economy has been steadily rising since 2004. The rate of increase from 2013 to 2014 slowed down slightly, and the rate of increase returned to the previous level after 2014. This is due to China's high emphasis on innovation. On the one hand, the government gave full play to the innovative leadership role of large enterprises, which led to the development of a group of innovative enterprises and technology-based SMEs with core competitiveness. Nowadays, some companies and industries have entered the top of the world, from chasers to leaders. On the other hand, the government encourages and supports enterprises to cooperate with schools and scientific research institutes; promotes the combination of production, education, and research; and provides a large number of innovative talents for various enterprises. At the same time, it promotes the reform of the innovation system and removes the system and mechanism barriers that restrict the vitality of innovation. These incentives for innovation are the key to the continuous improvement of China's innovation capabilities and are also an important part of the steady improvement of the top-notch growth of China's real economy.

## 4. The Experiment of Reducing Taxes and Fees on the High-Quality Development of the Real Economy

### 4.1. Policy Research Experiment on Tax and Fee Reduction

It examines the impact tax and fee waivers on the financial management of small and medium-sized enterprises by issuing questionnaires. From the perspective of enterprises, this paper explores the compatibility tax and fee waivers with the needs of enterprises. This paper selects 100 small- and medium-sized enterprises to carry out a questionnaire survey. It distributed 100 questionnaires and recovered 100 questionnaires, with a recovery rate of 100%. Among them, there are 69 valid questionnaires, accounting for 69% of the total questionnaires issued. The industries of the companies participating in the questionnaire are shown in Table 1:

It can be seen from Table 1 that among the valid questionnaires, there are 14 medium-sized enterprises (accounting for 20.29%) and 55 small enterprises (accounting for 79.71%). There are 60 general taxpayers (86.96%) and nine small-scale taxpayers (13.04%). The distribution of the annual tax payment scale of the enterprises participating in the questionnaire is shown in Figure 8:

Enterprises with an annual tax payment of less than 100,000 yuan (including 100,000 yuan) accounted for 31.88%, and enterprises with an annual tax payment of less than 100,000 to 500,000 yuan (including 500,000 yuan) accounted for 27.54%. Enterprises with an annual tax payment of less than 500–5 million yuan (including 5 million yuan) accounted for 28.99%, and enterprises with an annual tax payment of more than 5 million yuan accounted for 11.59%.

At present, under the influence of tax and fee reduction policies, the financial management of small- and medium-sized enterprises has more obvious shortcomings. Its management level will directly affect the implementation effect of preferential policies [26, 27].

The financial management of SMEs is affected by the tax and fee reduction policies. The questionnaire designed a question and six options for financial management issues that affect the policy of cutting tariff and costs. The options are that the management concept is not scientific enough, the management system is not standardized enough, the management objectives are not clear enough, the quality of financial personnel needs to be improved urgently, the internal control mechanism for financial management is lacking, and others. The financial governance problems that affect delivery tax and weight reduction policies are shown in Figure 9:

As can be seen from Figure 9, the companies participating in the survey believe that the first five options are all financial management issues that affect the enforcement of a policy to lower tuition and reduce fees, but the degree of recognition is slightly different. (1) The financial management concept is not scientific enough. Philosophy is a potential cultural force, and financial management concepts influence and even control the management practices of enterprises. Generally speaking, the financial management goal of an enterprise is to serve the goal of creating wealth or value for the enterprise. The scientific management concept will contribute to the current performance and future development of the enterprise; (2) The financial management system is not standardized enough [28, 29]. The financial management system is the system of the relationship between rights, responsibilities and interests in the financial management of enterprises. (3) The purpose of financial management is not clear enough. The purpose of enterprise financial management is the starting point and target point of all activities of the enterprise. (4) The quality of financial personnel needs to be improved urgently. Most of the financial staff stay at the level of “general understanding” of the tax and fee reduction policies closely related to their work content. This set of data directly reflects the urgent need to improve the quality of financial personnel. (5) Lack of internal control mechanism for financial management. Internal control mechanism is indispensable in modern economic management and supervision. It plays a vital role in improving the accuracy and reliability of accounting information. It involves many aspects such as corporate capital activities, procurement business, asset management, sales business, financial statements, and so on.

The results of the questionnaire showed that 44.83% of the respondents chose “lack of financial management internal control mechanism,” which is the same proportion as “lack of standard financial management system.” This shows that the respondents believe that the internal control mechanism of corporate financial management is as important as the financial management system.

### 4.2. Experiments for High-Quality Development of the Real Economy

Referring to the comprehensive index evaluation model method, this paper empirically measures the high-quality economic development level of China as a whole and 31 provinces (cities and regions) from 2010 to 2017. This is based on the sequence of China's high-quality economic development index and its subordinate five-dimensional index, as well as the economic top-notch growth index of 31 provinces (cities and regions) and its subordinate five-dimensional index sequence.

The specific processing method is as follows: (1) It is standardized according to the index. It forwards or reverses each indicator according to the specific meaning of the indicator and its theoretical meaning; (2) It calculates the information entropy of normalized data. If the information entropy of the indicator is larger, it means that the amount of information provided by the indicator is larger, and it should play a larger role in the comprehensive evaluation, and the weight should be higher. Information gauges the system's level of order and disorder is captured by using entropy; (3) It calculates the weight of each specific indicator through information entropy. As an objective weighting method, entropy weight method can deeply reflect the distinguishing ability of indicators and then determine the weight; (4) It calculates the indices of various dimensions of high-quality economic development through the index weights; (5) It obtains the high-quality economic development index through the summation of various dimension indices and equal weights [30–31]. The innovation and coordination index of top-notch growth of China's dimensional economy is shown in Table 2:

It can be seen from Table 2 that China's innovation achievements are remarkable, and the innovation index is rising year by year. Scientific and innovative has already emerged as an important force and a sharp weapon to promote national development and safeguard national security. The quality of coordination in China is improving, and the coordination index is generally rising. On the one hand, regional coordination has been strengthened. With the emphasis on urban and rural development, a new urban and rural economic and social integration development model is gradually taking shape. In the context of urbanization, the urbanization rate of household registration reached 43.4% in 2018. With the acceleration of industrialization and urbanization, the urban network system has been continuously improved. The number of cities increased from 132 in 1949 to 672 in 2018. In 2018, 99.5% of rural household-registered natural villages had access to roads, electricity, and telephones. More than 98% are able to receive cable TV signals, and more than 95% have broadband connections. On the other hand, the economic structure has been optimized. Agricultural production conditions have been greatly improved, and the industrial system has been gradually improved. Its ability to meet service demands improves. The industrial structure has changed from relying on one industry for development to relying on the common development of three industries. In 2018, the proportions of the primary, secondary, and tertiary industries were 7.2%, 40.7%, and 52.2%, respectively, and their contribution rates to economic growth were 4.2%, 36.1%, and 59.7%, respectively. The green and development index of top-notch growth of China's dimensional economy is shown in Table 3:

It can be seen from Table 3 that China's green development has risen in steps, and the effect of environmental governance has initially appeared. The overall increase in the degree of openness fluctuated significantly. According to data from the General Administration of Customs, in the first half of 2019, more than 5,000 customs-registered enterprises were added to the 12 free trade zones already in operation, bringing the total number of customs-registered enterprises to more than 85,000. Statistics from the Ministry of Commerce show that the total import and export volume reached 1.61 trillion yuan. It increased by 4.3% year-on-year, accounting for 10.97% of the total foreign trade in the same period (14.67 trillion yuan, a year-on-year increase of 3.9%). In terms of attracting foreign investment, the free trade zone achieved rapid growth, with the actual foreign investment increasing by 20.1% year-on-year, accounting for 14.5%. The top-notch growth and sharing of China's dimensional economy and the high-quality economic development index are shown in Table 4:

It can be seen from Table 4 that China's sharing index is increasing year by year, and the development of sharing is good. The achievements of China's economic aggregate have attracted worldwide attention. At the same time, there have been significant improvements in residents' income, social security, and quality of life. In 2018, the rural poor population dropped to 16.6 million, and the rural poverty rate dropped to 1.7%. Compared with 2012, it decreased by 82.39 million, which was 8.5% points lower than that in 2012. However, there is still room for improvement in supporting the general population in terms of compulsory education, medical care, and pensions. It also hopes to continue to provide substantive assistance to people in special difficulties and those in urgent need of assistance and draw a “bottom line” for the lives of the people.

## 5. Conclusions

As the material foundation of a country's economic and social development, the real economy plays a decisive role in the operation and development of the entire national economy. The development quality of the real economy is one of the decisive factors for whether China's economy can achieve top-notch growth. The high-quality development of China's economy is inseparable from the top-notch growth to the real economy. In today's world, with the continuous advancement of digital technology, the connection between the digital economy and the real economy is getting closer and closer. The digital economy has also been mentioned many times in important meetings and reports of the Chinese government. The tax reduction and fee reduction of big data algorithms have a positive effect on the top-notch growth of the real economy. It is necessary to vigorously develop the digital economy and cultivate high-quality talents to solve the problem of “stuck neck” in cutting-edge industries. It is necessary to accelerate the promotion of policy recommendations and contribute to the realization of top-notch growth of the real economy. Research on the impact of tax reduction and fee reduction based on big data algorithms on the high-quality development of the real economy is also of great significance for promoting current social development.

## Figures and Tables

**Figure 1:** The process of cluster analysis.

**Figure 2:** Spark architecture diagram.

**Figure 3:** Schematic diagram of KDD process.

**Figure 4:** Data mining analysis framework.

**Figure 5:** Tax revenue as a share of GDP.

**Figure 6:** The high-quality development trend of China's real economy over the years.

**Figure 7:** Trends of China's real economy innovation indicators over the years.

**Figure 8:** Distribution of annual tax payment scale of enterprises.

**Figure 9:** Financial management issues that affect the effect of tax and fee reduction policies.

**Table 1:** Statistical table of the industry to which the enterprise belongs.

Enterprise	Subtotal	Proportion
Agriculture, forestry, animal husbandry and fishery	0	0%
Industry	10	14.49%
Construction	3	4.35%
Wholesale industry	11	15.94%
Retail	10	14.49%
Communications and transportation industry	0	0
Storage industry	1	1.45%
Postal industry	0	0
Accommodation industry	1	1.45%
Catering	1	1.45%
Information transmission industry	1	1.45%
Software and information technology services	5	7.25
Real estate development and operation	1	1.45
Estate management	6	8.69
Leasing and business services	7	10.14
Other	12	17.39
Total	69	

**Table 2:** Innovation and coordination index of high-quality development of China's dimensional economy.

Particular year	Innovation index	Coordination index
2010	0.02833463	0.38927972
2011	0.18260529	0.40299964
2012	0.28650363	0.48126008
2013	0.4135686	0.51537136
2017	0.47167973	0.49224842
2015	0.62569894	0.55697941
2016	0.70598714	0.51717563
2017	0.96430399	0.49194163

**Table 3:** Green and development index of high-quality development of China's dimensional economy.

Particular year	Green index	Development index
2010	0.15510578	0.36015677
2011	0.27841842	0.45615397
2012	0.36012129	0.48513864
2013	0.67605050	0.35046657
2017	0.75270730	0.36244286
2015	0.75768333	0.44101034
2016	0.78902400	0.51234636
2017	0.8386	0.68936552

**Table 4:** China's dimensional economic high-quality development sharing and economic high-quality development index.

Particular year	Sharing index	High-quality index
2010	0.03808856	0.19419309
2011	0.21372841	0.30678115
2012	0.35419119	0.39344296
2013	0.49967016	0.49102563
2017	0.62632785	0.54108123
2015	0.73439365	0.62315314
2016	0.81256550	0.66741973
2017	0.93416832	0.78387587

## Data Availability

Data sharing is not applicable to this article as no new data were created or analyzed in this study.
